# Study on Psychological Stress Response and Intervention Countermeasures of Exposed Population under Sudden Public Health Crisis

**DOI:** 10.1155/2022/3411960

**Published:** 2022-07-25

**Authors:** Si Chen, Hongwei Sun, Min Zhang, Jihong Wang, Yan Song, Chunshan Zhao, Lei Zhou, Yali Sun, Qinlan Lin, Changping Song, Yanchun Gu, Shengnan Wang

**Affiliations:** ^1^Wei Fang Medical University, Weifang City, Shandong 261053, China; ^2^Bei Hua University, Jilin City, 132013, China; ^3^China CDC, 102206, China

## Abstract

**Background:**

After the occurrence of public health emergencies, people will have a series of physiological reactions, which will develop into psychological stress disorder in serious cases. Based on this, the purpose of this study is to analyze the psychological stress response and intervention countermeasures of exposed people under sudden public health crisis.

**Objective:**

To explore the psychological stress response and intervention countermeasures of exposed population under sudden public health crisis.

**Methods:**

A total of 400 people under the sudden public health crisis that bring about serious damage to public health, mass diseases of unknown causes, major food and occupational poisoning, and other events that seriously affect public health from December 2020 to December 2021 were selected as the subjects of the study. It was randomly and equally divided into two groups to take different intervention measures, the control group was given routine public health crisis intervention measures, and the research group was given comprehensive intervention. The metabolism, social function defects, health symptoms, psychological status, quality of life, sleep quality, and stress reaction were compared between the two groups.

**Results:**

The rate of good metabolism in the research group was significantly higher than that in the control group (*P* < 0.05). After intervention, the scores of Social Disability Screening Schedule (SDSS) and Symptom Checklist 90 (SCL-90) decreased in both groups, and the scores of SDSS and SCL-90 in the research group were lower than those in the control group. After intervention, the scores of self-rating depression scale and self-rating anxiety scale in the two groups decreased, and the scores of self-rating depression scale and self-rating anxiety scale in the research group were lower than those in the control group (*P* < 0.05). The sleep quality of the research group was better than that of the control group (*P* < 0.05). The stress response indexes such as cortisol, blood glucose, and C-reactive protein in the two groups were decreased after intervention. The stress response indexes such as cortisol, blood glucose, and C-reactive protein in the research group were lower than those in the control group (*P* < 0.05).

**Conclusion:**

Giving that comprehensive intervention measures to people exposed to sudden public health crisis can effectively relax their stress response, reinvigorate their quality of life and sleep, reduce depression and anxiety, and improve their metabolism, therefore, in the case of the outbreak of public health crisis in the future, it is worth applying for reference and popularizing.

## 1. Introduction

Public health emergency refers to the sudden occurrence of major infectious diseases that bring about serious damage to public health, mass diseases of unknown causes, major food and occupational poisoning, and other events that seriously affect public health [1–4]. In the International Health Regulations adopted in 2005, an international public health emergency is defined as an unusual event that poses a public health risk to other countries through the international spread of the disease and may require a coordinated international response [5]. The international public health emergency was first put forward by the World Health Organization (WHO) and recognized by the health systems of all countries in the world [6]. It is proposed to prevent and reduce the spread of diseases on the one hand and reduce the interference to the international economy and traffic on the other hand when dealing with global public health events. Public health emergencies will elicit serious damage to people's mental psychology [7, 8]. Previous studies have shown that about half of people may have been exposed to traumatic events [9, 10]. After the occurrence of public health emergencies, people will have a series of physiological reactions, which we call stress reactions, and in serious situation, they will develop into psychological stress disorders. With the continuous development of stress research, more and more scholars begin to pay attention to the role of psychosocial factors in stress and find that coping style, social support, and personality characteristics play an important role in psychological stress [11–14]. Based on this, the purpose of this study is to analyze the psychological stress response and intervention countermeasures of the exposed population under the sudden public health crisis, and the process and results are reported as follows.

## 2. Materials and Methods

### 2.1. General Information

A total of 400 people under the sudden public health crisis from December 2020 to December 2021 were selected as the object of study. It was randomly divided into two groups to take different intervention countermeasures. In the control group, the age was 23-74 years old, with an average of 45.91 ± 3.63 years, including 108 males and 92 females, while in the research group, the age was 24-76 years old, with an average of 45.96 ± 3.58 years, including 104 males and 96 females. The general data of the two groups were not statistically significant. All the people signed informed consent. This study was a double blind test.

Recruiting criteria are as follows: (1) age ≥ 18 years old; (2) good communication skills and no language barrier and can actively cooperate with relevant scores, examinations, and inquiries; and (3) vital signs are stable.

Exclusion criteria re as follows: (1) with severe heart, liver, renal insufficiency, malignant tumors, and other diseases; (2) patients with long-term infection or short-term infection were not cured after treatment; and (3) patients with serious compound injuries such as the head, abdomen, spine, and limbs.

### 2.2. Intervention Methods

The control group was given routine intervention measures, including psychological counseling and health education. The research group was given comprehensive intervention measures: (1) Positive self-regulation. In the face of public health emergencies, we should learn to carry out positive self-regulation through internal and external regulation. Internal regulation is to change one's own cognitive model and coping behavior model, so as to change the emotional state. Cognitive behavioral therapy believes that the cognitive process determines the generation of behavior and emotional changes. Therefore, cognitive reconstruction should be carried out to identify individual unreasonable beliefs and actively seek change. External adjustment is to adjust the psychological state with the help of external forces, such as adjusting interpersonal relations, obtaining social support, and solving problems. (2) Receptive emotion. Knowing and accepting one's emotions is the basis of learning to manage emotions. When negative emotion occurs, if you try to fight it, it will only occupy more cognitive resources and make it more distracting and unable to focus on what you want to do. Therefore, instead of immersing in negative emotion, we should learn to accept emotion, try to feel its existence when negative emotion appears, acknowledge its inevitability, and use its message to make a more rational, complete and realistic judgment. (3) Strengthen the interaction with the outside world. During public health emergencies, prolonged home isolation can lead to anxiety, depression, and insecurity. We should strengthen contact with the outside world, get in touch with friends, classmates and teachers, and share personal views, so as to maintain connection and interaction with the outside world and alleviate personal negative emotions. (4) Aerobic exercise. When an individual is doing aerobic exercise, the heart pressure will increase, and the brain will make the judgment of fighting or running away, and then release brain-derived neurotrophic factor, which can protect and repair memory neurons. At the same time, the brain releases endorphins. Endorphins, known as “happiness stimuli,” can minimize discomfort caused by exercise, reduce pain, and make people feel excited. During public health emergencies, we can regulate our emotions through indoor aerobic exercise, such as aerobics, running in place, and rope skipping. (5) Perfect the three-level work system of psychological counseling. Good psychological counseling should not only solve the current problems of visitors but also make them achieve spiritual growth and help them acquire the ability to solve similar problems. In order to achieve this goal, professional psychological counselors should be selected, the working mechanism of online psychological counseling should be improved, and the three-level work system should be implemented. The first level is online intervention, the intervention content is the direct psychological stress response caused by public health emergencies, nd counselors can provide online help within 30 minutes. On this basis, if visitors are found to have physical discomfort or past psychological problems caused by public health emergencies, they should enter the second-level intervention and other counselors will provide them with psychological counseling for more than 30 minutes. Among such visitors, if the counselor finds that there are visitors who need long-term follow-up, they will enter the third-level intervention and should provide them with continuous psychological support after seeking the consent of the supervisor until the problem is solved.

### 2.3. Observation Index

#### 2.3.1. Metabolic Assessment

The body weight, waist circumference, fasting blood glucose, systolic blood pressure, diastolic blood pressure, fasting triglyceride, and fasting high-density lipoprotein were measured before and after intervention. Good: the above indicators have significantly improved and basically returned to the normal level; in general: the above indicators have slightly improved compared with the preintervention, but still worse than the normal level; poor: do not meet the good and general evaluation criteria. Good rate = (good + average)/number of cases∗100%.

#### 2.3.2. Evaluation Methods of Social Functional Defects and Health Symptoms

The social disability function of the people was evaluated by the Social Disability Screening Scale (SDSS) [15]. The scale was evaluated in terms of occupation and work, parental functions, social withdrawal, social activities outside the family, too few activities within the family, family functions, personal self-care, interest and concern for the outside world, responsibility and planning, etc. each item was rated as 0.1 and 2 points, with 0 as normal or with only minor defects. 1 is that there is a real functional defect, and 2 is that there is a serious functional defect. The second and third items of the unmarried were not included in the total score, and the higher the score, the more serious the overall social function defect of the patients.

Symptom Checklist 90 (SCL-90) [16] was used to evaluate the health status of the two groups before and after intervention. The scale is divided into 10 categories and 90 items, such as somatization, obsessive-compulsive disorder, interpersonal sensitivity, depression, anxiety, hostility, phobia, paranoia, and mental illness (reflecting sleep and diet). Item scoring system: according to the degree of symptom, the scores of mild, moderate, severe and severe was 1-5 points, respectively. The higher the score, the worse the health.

#### 2.3.3. Evaluation Method of Mental State before and after Intervention

The Self-Rating Depression Scale (SDS) [17] was used to evaluate the depression state of parturients before and after intervention: the scale contained 20 items reflecting the subjective feelings of depression, and each item was divided into four grades according to the frequency of symptoms, of which 10 were positive scores and 10 were reverse scores. The cut-off value of the SDS standard score was 53, of which 53-62 was mild depression, 63-72 was moderate depression, and more than 73 was severe depression.

The Self-Rating Anxiety Scale (SAS) [18] was used to evaluate the anxiety state of parturients before and after intervention: SAS used 4 grades, which mainly assessed the frequency of symptoms defined by the item, the criteria were as follows: “1” no or little time, “2” a small part of time, “3” a considerable amount of time, and “4” most or all of the time. It is normal for people with an overall anxiety score below 50. Those with a score of 50-60 are mild, those with a score of 61-70 are moderate, and those with a score of 70 or more are severe anxiety.

#### 2.3.4. Evaluation Methods of Quality of Life and Sleep Quality

The SF-36 Health Survey Scale [19] was used to analyze the quality of life of the two groups after nursing, including physiological function, physiological function, emotional function, social function, vitality, physical pain, mental health, general health 8 dimensions; a total of 36 items, each item 0-6 points, take the average score; the higher the score, the better the quality of life of the patients.

The Pittsburgh Sleep quality Index (PSQI) [20] was used to evaluate the sleep quality of parturients after intervention with different nursing management modes. The scale consists of 18 items and 7 components, including falling asleep time, sleep quality, sleep efficiency, sleep disorders, sleeping drugs, and daytime function. Each component is scored according to the 0 : 3 grade, the cumulative score of each component is the total score of PSQI, the total score range is 0 : 21; the higher the score, it means the worse the quality of sleep.

#### 2.3.5. Comparison of Stress Response Indexes between the Two Groups

Fasting blood samples were collected on the first day before operation and the first day after operation, and the levels of serum cortisol, blood glucose, and C-reactive protein were measured. C-reactive protein was determined by latex enhanced scatter immunoturbidimetry and Abbott C8000 automatic biochemical instrument.

### 2.4. Statistical Analysis

We used SPSS 21.0 statistical software for statistical analysis. The measurement data were expressed in $\bar{x}\pm s$, and the normal distribution and homogeneity of variance were tested before statistical analysis. *t*-test was used to compare the two groups of measurement data, *n* (%) was used to represent the counting data, and *χ*^2^ test was used for statistical analysis. The difference was statistically significant (*P* < 0.05).

## 3. Results

### 3.1. Comparison of Metabolism Status

In the comparison of metabolism between the two groups, 109 cases were good, 80 cases were general, 11 cases were poor, and the rate of good metabolism was 94.5%. In contrast, in the control group, 100 cases were good, 76 cases were general, 24 cases were poor, and the rate of good metabolism was 88%. The rate of good metabolism in the research group was higher than that in the control group, and the difference was statistically significant (*P* < 0.05). The above results show that the therapeutic effect of the research group is better than that of the control group. All the data are shown in Figure 1.

### 3.2. Comparison of SDSS Score and SCL-90 Score before and after Intervention

Before the intervention, there was no significant difference in the SDSS score and SCL-90 score between the two groups, but after the intervention, the SDSS score and SCL-90 score of the two groups decreased, and the SDSS score and SCL-90 score of the research group were lower than those of the control group, and the difference was statistically significant (*P* < 0.05). The above results show that the therapeutic effect of the research group is better than that of the control group. All the data are shown in Figure 2.

### 3.3. Comparison of SDS and SAS Scores before and after Intervention

In terms of the scores of SDS and SAS, there was no significant difference between the two groups before intervention, but after intervention, the scores of SDS and SAS of the two groups decreased, and the scores of SDS and SAS of the research group were lower than those of the control group, and the difference was statistically significant (*P* < 0.05). The above results show that the therapeutic effect of the research group is better than that of the control group. All the data are shown in Table 1.

### 3.4. Comparison of SF-36 Scores after Intervention

After intervention, the SF-36 scores of physiological function, emotional function, social function, vitality, physical pain, mental health, and overall health in the research group were significantly higher than those in the control group (*P* < 0.05). The above results show that the therapeutic effect of the research group is better than that of the control group. All the data are shown in Table 2.

### 3.5. Comparison of Sleep Quality after Intervention

After the intervention, the sleep quality of the two groups was compared, and the scores of falling asleep time, sleep quality, sleep efficiency, sleep disorders, sleeping drugs, and daytime function in the research group were lower than those in the control group (*P* < 0.05). The difference was statistically significant (*P* < 0.05). The above results show that the therapeutic effect of the research group is better than that of the control group. All the data are shown in Table 3.

### 3.6. Comparison of Stress Response Indexes before and after Intervention

Before intervention, there was no significant difference in stress response indexes such as cortisol, blood glucose, and C-reactive protein between the two groups (*P* > 0.05). After intervention, the stress response indexes such as cortisol, blood glucose, and C-reactive protein in the two groups were decreased, but compared with the control group, the stress response indexes such as cortisol, blood glucose, and C-reactive protein in the research group were lower than those in the control group; the differences were statistically significant (*P* < 0.05). The above results show that the therapeutic effect of the research group is better than that of the control group. All the data are shown in Table 4.

## 4. Discussion

In recent years, major public health emergencies have emerged one after another, such as terrorist attacks, tsunamis, the spread of SARS and avian influenza, and the global pandemic of COVID-19 since 2019. Public health emergencies will not only lead to economic losses and political instability but also exert serious harm to people's mental health [21]. Public health emergencies have the following characteristics: diversity of causes, differences in distribution, widespread transmission, complexity of hazards, comprehensiveness of governance, continuous emergence of new events, diversity of types, foodborne diseases and food poisoning are easy to appear and will also bring serious consequences, and public health events occur frequently [22]. Previous studies have shown that about 50% or 70% of people may have been exposed to traumatic events in their lifetime [23]. After the occurrence of public health emergencies, people will appear with a series of psychological and physiological reactions, which we call stress reactions, and in serious cases, they will develop into stress disorders. In different stress states, there can be different intensity of physiological reactions. The regulation of these responses depends on the body's neural, immune, and endocrine systems [24]. These physiological reactions can make the body recover from the disorder induced by stress as much as possible through the feedback mechanism to each system. In the face of stress, this is the adaptation process of the body, and it may also be responsible for psychosomatic diseases.

In this study, compared with the metabolism of the two groups, 109 good, 80 general, and 11 poor people were found in the research group, and the rate of good metabolism was 94.5%. The rate of good metabolism in the control group was 100 cases, 76 cases, and 24 cases, respectively. The rate of good metabolism was 88%. Compared with the control group, the rate of good metabolism in the research group was higher than that in the control group (*P* < 0.05). The analysis shows that under stress, people's metabolism may be reduced, and effective intervention strategies can significantly improve the metabolic capacity of exposed people under public health emergencies and avoid diseases caused by impaired metabolic function. Fear refers to a feeling of tension and worry in the face of a threat and cannot get rid of it. Individuals are often accompanied by avoidance behavior while producing fear in order to avoid danger. Anxiety is an unpleasant experience of an individual to an event that may result in danger. Anxiety often has physiological and behavioral reactions such as flutter, sweating, dry mouth, and rubbing hands back and forth [25]. According to the results of our study, after intervention, the scores of SDS and SAS in both groups decreased. The scores of SDS and SAS in the research group were significantly lower than those in the control group. The analysis uncovered that comprehensive intervention helps to reduce the level of anxiety and depression in patients.

In this study, there was no significant difference in the SDSS score and SCL-90 score between the two groups before intervention, but after intervention, the SDSS score and SCL-90 score of the two groups decreased, and compared with the control group, the SDSS score and SCL-90 score of the research group were lower than those of the control group. Studies have shown that long-term sleep disorders can increase blood pressure; increase metabolism, cardiovascular system function, and neurological disorders; and then aggravate the state of psychological stress [25]. Anxiety and depression can increase sympathetic tension and catecholamine secretion and make the body produce physical discomfort symptoms such as palpitation, chest tightness, muscle tension, and even near-death feeling, which become the main causes affecting sleep, and at the same time, it can also increase psychological burden and aggravate adverse emotions and stress reactions [25]. After the intervention, the sleep quality of the two groups was compared, and the scores of falling asleep time, sleep quality, sleep efficiency, sleep disorders, sleeping drugs, and daytime function in the research group were lower than those in the control group. The analysis shows that the stronger the unpredictability and uncontrollability of stress events, the stronger the psychological stress reaction and the more serious the physiological disorder, which can easily affect the quality of life and sleep effect of the people. However, if individuals have a certain degree of understanding of stress events before they occur and take appropriate strategies to intervene, they can relatively alleviate psychological and physical stress reactions, thus improving the quality of life and sleep effect.

Some studies have shown that cortisol affects the activation of the hypothalamus-pituitary adrenal axis by stress, which leads to changes in glucocorticoid secretion and weight loss, depression, and anxiety-like manifestations such as reduced activity [26–28]. The main manifestations are increased excitability of hypothalamus-pituitary-adrenocortical axis and increased secretion of glucocorticoids, in which cortisol is the main glucocorticoid in human body. The level of plasma cortisol during stress reflects the degree of stress response. Moderate stress response is beneficial to the human body and helps the body to quickly adapt to the internal and external environment. Cortisol is a stress hormone closely related to the metabolic system, which increases the body's resistance [27]. Cortisol is a sensitive index to reflect the stress response of the body. The stimulation of adverse factors can promote the secretion of adrenocortical hormone, and the increase of plasma cortisol during stress is rapid and significant. After physical and mental trauma, cortisol secretion is at its peak and relatively stable. As an index of stress metabolic response, blood glucose tends to be stable with cortisol secretion after trauma intervention. Therefore, the stress status can be evaluated by cortisol, blood glucose, and other stress indexes. Inflammatory reaction is another form of stress reaction [29]. C-reactive protein is a kind of inflammatory factor, and its expression can be significantly increased in a short time after tissue injury. Combined with the results of this study, there was no significant difference in stress response indexes such as cortisol, blood glucose, and C-reactive protein between the two groups before intervention (*P* > 0.05). After intervention, the stress response indexes such as cortisol, blood glucose, and C-reactive protein in the two groups decreased. Compared with the control group, the stress response indexes such as cortisol, blood glucose, and C-reactive protein in the research group were significantly lower than those of the control group. The analysis indicates that the stress response is a kind of nonspecific response after the body is stimulated by external trauma and various factors. When trauma occurs, the hypothalamus-pituitary-adrenal cortex axis and sympathetic-adrenal medulla system are activated, secreting large amounts of cortisol, resulting in fat mobilization and insulin resistance, and increasing blood sugar. Cortisol is an important substance to maintain the stability of the environment in the body, and its plasma content is positively correlated with the duration and intensity of stimulation [29]. These physiological changes provide sufficient preparation for the body to cope with external stimuli. In the short term, these reactions are conducive to the adaptation of the body to external stimuli; if the stimulation duration is too long or the intensity is too large, the body can be exhausted, resulting in autonomic nervous dysfunction, resulting in a variety of physical and psychological disorders [29]. The same idea can be found in the study put forward by Wang [30]. They have applied new methods in the study, and the conclusions drawn can also give some support to this study.

Collectively, giving that comprehensive intervention measures to people exposed to sudden public health crisis can effectively relax their stress response, reinvigorate their quality of life and sleep, reduce depression and anxiety, and improve their metabolism; therefore, in the case of the outbreak of public health crisis in the future, it is worth applying for reference and popularizing.

## Figures and Tables

**Figure 1:** Comparison of metabolism between the two groups.

**Figure 2:** Comparison of the SDSS score and SCL-90 score before and after intervention Note: compared with before intervention, a: *P* < 0.05; compared with the research group, b: *P* < 0.05.

**Table 1:** Comparison of SDS and SAS scores before and after intervention ($\bar{x}\pm s$, points, *n* = 200).

Group	SDS		SAS	
	Before intervention	After intervention	Before intervention	After intervention
Control group	45.63 ± 5.12	41.45 ± 4.36^a^	43.56 ± 5.74	38.82 ± 5.44^a^
Research group	45.46 ± 5.14	27.76 ± 3.28^b^	43.17 ± 5.56	29.48 ± 5.23^b^
*t*	0.331	35.485	0.690	17.504
*P*	0.741	0.000	0.491	0.000

Note: the control group before and after intervention, ^a^*P* < 0.05; the research group before and after intervention, ^b^*P* < 0.05.

**Table 2:** Comparison of SF-36 scores between the two groups after intervention ($\bar{x}\pm s$, points, *n* = 200).

Group	Physiological function	Emotional function	Social function	Vitality	Somatic pain	Mental health	Overall health
Control group	74.31 ± 5.14	75.02 ± 6.72	73.46 ± 5.23	72.64 ± 5.92	73.15 ± 5.62	72.71 ± 6.31	74.34 ± 6.20
Research group	82.46 ± 5.40	86.32 ± 6.91	85.67 ± 5.42	82.15 ± 6.14	85.28 ± 6.22	83.38 ± 5.89	82.51 ± 7.17
*t*	15.460	16.579	22.926	15.769	20.464	17.481	12.189
*P*	0.000	0.000	0.000	0.000	0.000	0.000	0.000

**Table 3:** Comparison of sleep quality between the two groups after intervention ($\bar{x}\pm s$, points, *n* = 200).

Group	Falling asleep time	Sleep quality	Sleep efficiency	Sleep disorder	Sleeping drug	Daytime function
Control group	2.14 ± 0.43	1.84 ± 0.42	2.58 ± 0.61	1.88 ± 0.87	1.98 ± 0.74	2.18 ± 0.28
Research group	1.33 ± 0.34	1.23 ± 0.53	1.54 ± 0.58	1.38 ± 0.66	1.38 ± 0.52	1.28 ± 0.31
*t*	20.897	12.757	17.473	6.475	9.382	30.469
*P*	0.000	0.000	0.000	0.000	0.000	0.000

**Table 4:** Comparison of stress response indexes between the two groups before and after intervention ($\bar{x}\pm s$, *n* = 200).

Group	Cortisol (ng/mL)		Blood sugar (mmol/L)		C-reactive protein (mg/L)	
	Before intervention	After intervention	Before intervention	After intervention	Before intervention	After intervention
Control group	93.41 ± 20.05	77.44 ± 23.30^a^	4.55 ± 1.58	3.55 ± 1.37^a^	26.46 ± 8.31	18.58 ± 4.11^a^
Research group	93.38 ± 20.11	61.82 ± 16.29^b^	4.43 ± 1.15	2.72 ± 1.10^b^	26.50 ± 8.42	13.37 ± 4.85^b^
*t*	0.015	7.770	0.768	6.681	0.048	7.069
*P*	0.988	0.000	0.444	0.001	0.962	0.000

Note: the control group before and after intervention, ^a^*P* < 0.05; the research group before and after intervention, ^b^*P* < 0.05.

## Data Availability

No data were used to support this study.
